The article "Evaluation of RNA Extraction-Free Method for Detection of SARS-CoV-2 in Salivary Samples for Mass Screening for COVID-19" was published in 2021. Journal: Biomed Res Int.

# Evaluation of RNA Extraction-Free Method for Detection of SARS-CoV-2 in Salivary Samples for Mass Screening for COVID-19

**DOI:** 10.1155/2021/5568350

**Published:** 2021-06-29

**Authors:** Sally A. Mahmoud, Subhashini Ganesan, Esra Ibrahim, Bhagyashree Thakre, Juliet G. Teddy, Preety Raheja, Walid Z. Abbas

**Affiliations:** ^1^Biogenix G42 Lab, Abu Dhabi, UAE; ^2^G42 Health Care, Abu Dhabi, UAE

## Abstract

In this COVID-19 pandemic, there is a dire need for cost-effective and less time-consuming alternatives for SARS-CoV-2 testing. The RNA extraction-free method for detecting SARS-CoV-2 in saliva is a promising option. This study found that it has high sensitivity (85.34%), specificity (95.04%), and was comparable to the gold standard nasopharyngeal swab (NPS) sample tests. The method showed good agreement between salivary and NPS samples, with a kappa coefficient of 0.797. However, there are variations in the sensitivity and specificity based on the RT-PCR kit used. The Thermo Fisher Applied Biosystems showed high sensitivity, positive predictive value (PPV), and negative predictive value (NPV) but also showed a higher percentage of invalid reports. On the other hand, the BGI kit showed high specificity, better agreement (kappa coefficient) between the results of saliva and NPS samples, and higher correlation between the Ct values of saliva and NPS samples. Thus, the RNA extraction-free method for salivary sample serves as an effective alternative screening method for COVID-19.

## 1. Introduction

The current pandemic caused by the SARS-CoV-2 virus, widely known as COVID-19, has affected more than 75 million people worldwide and, as of 20th December 2020, has caused more than 1.6 million deaths according to the WHO [1]. Early identification, isolation, and contact tracing play a vital role in controlling the pandemic. The high number of COVID-19 cases and transmissibility of the virus warrants mass screening, which involves a large number of diagnostic tests to be conducted. Currently, sample collection with nasopharyngeal swabbing followed by RT-PCR is the gold standard for diagnosis of COVID-19 [2].

Nasopharyngeal swabs have multiple limitations. They require trained personnel to collect the sample; there is a risk of exposure for the healthcare personnel procuring the sample, and there is discomfort to the patients during the procedure. There are also contraindications for performing nasopharyngeal swabbing, such as coagulopathies, anticoagulant therapy, and deviated nasal septum. Moreover, when the swabbing is performed incorrectly, an adequate sample might not be obtained, leading to inconclusive or invalid results and the need to repeat swabbing. This method of sample collection also requires the use of personal protective equipment (PPE) by the healthcare personnel collecting the swab, as there is a high risk of exposure, leading to additional drain on resources. All the abovementioned aspects suggest the need for alternative methods of testing and diagnosis for COVID-19; saliva seems to be an excellent available alternative.

The article "Evaluation of RNA Extraction-Free Method for Detection of SARS-CoV-2 in Salivary Samples for Mass Screening for COVID-19" was published in 2021. Journal: Biomed Res Int.

The human saliva has hundreds of microbial species, many of which are related to diseases affecting humans [3], including hereditary diseases, autoimmune diseases, malignancies, and infections [4, 5]. Saliva has also been used as an important diagnostic tool in previous coronavirus infections like Severe Acute Respiratory Syndrome (SARS) and Middle East Respiratory Syndrome (MERS) [6].

Diagnosis of viral infections from salivary samples depends on various factors, including the presence of the virus in the saliva, viral load, and quantities of particles like DNA, RNA, antigens, and host antibodies [7, 8]. The duration and stage of infection are also important as some viruses can be detected in saliva almost a month after infection [7, 8].

In the context of COVID-19, the saliva plays a crucial role in the transmission of the disease, as droplets are the main source of human-to-human transmission. The saliva contains the viral particles, anti-SARS-CoV-2 antibodies, and infected host cells, which can be used for diagnostic, as well as prognostic, purposes [9, 10]. Further, the infection of salivary glands occurs earlier in the disease course for COVID-19 [11]. The viral load in saliva is highest during the first week of onset, and viral particles can be detected in saliva up to 25 days after the onset of infection. This suggests saliva as an effective, noninvasive alternative method for diagnosis of COVID-19 [12].

Saliva testing offers additional advantages when mass testing is required, as it is noninvasive and does not require a trained healthcare personnel to collect the sample. This alleviates the need for PPE, swabs, and other materials, allowing for increased access for other areas in need. Additionally, there is reduced-to-no risk of exposure for the health personnel, as the individual patient can collect the sample. On top of this, there are no contraindications for this method of sample collection; it is more comfortable for patients, especially when multiple tests are performed, and salivary samples allow for other types of disease monitoring [11–13].

This study is aimed at exploring how efficient RNA extraction-free method is for detection of SARS-CoV-2 in saliva, as an alternative specimen for COVID-19 testing.

### 1.1. Objectives

1. To compare the sensitivity and specificity of the RNA extraction-free method for molecular testing of SARS-CoV-2 of salivary sample versus nasopharyngeal samples
2. To compare the efficiency of RNA extraction-free method for SARS-CoV-2 detection on salivary samples using BGI Genomics' 2019-nCoV Fluorescence Detection Real-Time RT-PCR kit and Thermo Fisher Applied Biosystems TaqPath COVID-19 CE-IVD RT-PCR kit

The article "Evaluation of RNA Extraction-Free Method for Detection of SARS-CoV-2 in Salivary Samples for Mass Screening for COVID-19" was published in 2021. Journal: Biomed Res Int.

## 2. Methodology

### 2.1. Sample Size Calculation

The SARS-CoV-2 infection positivity was around 5% in our lab at the time of the study. With the recommendation based on Bujang et al. [14], we calculated the minimum sample size to be 380 participants, including 19 positive cases to achieve a minimum power of at least 80%, at a significance level of 5%, to detect a sensitivity of 95%. This sample would also be able to detect a specificity of 95%.

### 2.2. Methods

The study was approved by the Department of Health (DOH) Institutional Review Board (IRB), Abu Dhabi. The study followed all regulations and guidelines of the IRB. The participants of the study were well-informed about the details of the study, and informed consent was obtained. After obtaining the consent, one nasopharyngeal swab (NPS) and one salivary sample were collected from each participant. A total of 600 people participated in the study. The NPS samples were collected by trained healthcare personnel, as per protocol in place, and were immediately transported to the lab. The salivary samples were collected in a sterile Dnase/Rnase-free container without any stabilizing agent. Instructions were given to all participants before saliva collection. The preconditions for saliva collection included no food, drink, smoking, nor oral hygiene products for at least one hour prior to sample collection. Participants were asked to pool saliva in his or her mouth for 1–2 minutes before depositing the salivary sample into a collection tube. The collected salivary samples were transported to the lab in temperature-controlled boxes at 2-8 degrees Celsius, where they were processed by a nucleic acid extraction-free method for SARS-CoV-2 detection.

### 2.3. RNA Extraction for the Nasopharyngeal Swabs

The nasopharyngeal swabs collected from participants were transported using viral transport medium (VTM). All methods were carried out in accordance with relevant guidelines and regulations. In the lab, RNA extraction was performed by the automated machine MGISP-960, as per the manufacturer's instructions. After the RNA extraction, 10 microliters of the sample extract was added to 20 and 15 microliters of the master mix for the BGI Genomics' 2019-nCoV Fluorescence Detection Real-Time RT-PCR kit and the Thermo Fisher Applied Biosystems TaqPath COVID-19 CE-IVD RT-PCR kit, respectively. Both the extraction and the PCR detection methods were verified in house. The real time fluorescent RT-PCR was performed using the Bioer LineGene 9600 Plus Fluorescent Quantitative Detection System for BGI Genomics' 2019-nCoV Fluorescence kit and on the QuantStudio 5 Real-Time PCR System machine for the Applied Biosystems TaqPath kit.

The article "Evaluation of RNA Extraction-Free Method for Detection of SARS-CoV-2 in Salivary Samples for Mass Screening for COVID-19" was published in 2021. Journal: Biomed Res Int.

### 2.4. RNA Extraction-Free Direct Method for Salivary Samples

It is a nucleic acid extraction-free method for SARS-CoV-2 detection following the protocol of Saliva-Direct test, a saliva-based, nucleic-acid-extraction-free, RT-qPCR method for SARS-CoV-2 detection [15]. 50 microliters of the salivary sample collected is used for the assay. The salivary sample is first treated with proteinase K, followed by a heat inactivation step, and is then directly used as input in the RT-PCR test using validated primer and probe sets (Figure 1). The RT-qPCR was performed using BGI Genomics' 2019-nCoV Fluorescence Detection Real-Time RT-PCR kit and Thermo Fisher Applied Biosystems kit.

### 2.5. The BGI Genomics' 2019-nCoV Fluorescence Detection Real-Time PCR Kit (BGI Kit) [16]

The Real-Time Fluorescent RT-PCR kit for detecting SARS-2019-nCoV is used for the identification of SARS-CoV-2 RNA in nasopharyngeal swabs, throat swabs, and Broncho Alveolar Lavage Fluid (BALF) from patients with SARS-CoV-2. The RT-qPCR procedure was performed following manufacturer's instructions and was optimized for processing saliva samples.

For optimization, results with high CT values for viral genes (ORF1AB) at FAM channel (CT value > 35 and ≤38) or with abnormal amplification curves were reprocessed for confirmation. Samples with CT values > 38 and S-shaped amplification curves are considered in the grey zone and were reprocessed for confirmation. If the same result was obtained with the repeat testing, the result was confirmed as positive. This optimization was done to avoid false positive results at higher CT values. For each test specimen, VIC must present “S” curve with VIC Ct value ≤ 32; when Ct values at VIC channels are higher than 32 or if there was no Ct value at VIC, the sample was considered invalid.

### 2.6. The Thermo Fisher Applied Biosystems TaqPath COVID-19 CE-IVD RT-PCR Kit (Thermo Fisher Kit) [17]

TaqPath COVID-19 CE-IVD RT-PCR kit contains the reagents and controls for Real-Time Reverse Transcription Polymerase Chain Reaction (RT-PCR) test intended for the qualitative detection of nucleic acid from SARS-CoV-2 in upper respiratory specimens (such as nasopharyngeal, oropharyngeal, nasal, and midturbinate swabs and nasopharyngeal aspirate) and bronchoalveolar lavage (BAL) specimens from individuals suspected of COVID-19. It is a multiplex assay that contain three primer/probe sets specific to different SARS-CoV-2 genomic regions and primers/probes for bacteriophage MS2. The manufacturer instructions were followed, and reporting was done as per the instructions. When all three genes ORFa1b, N, and S are negative and MS2 (blank control) gene is also negative, then the test is termed invalid.

The article "Evaluation of RNA Extraction-Free Method for Detection of SARS-CoV-2 in Salivary Samples for Mass Screening for COVID-19" was published in 2021. Journal: Biomed Res Int.

To compare the efficiency of RNA extraction-free method of salivary sample in RT-qPCR-based testing with BGI RT-PCR kit and Thermo Fisher Applied Biosystems RT-PCR kit, 258 random samples out of the 600 salivary and NPS were processed through the RT-qPCR machine using the Thermo Fisher Applied Biosystems kit. The reports of the salivary sample processed through both these kits were compared with the results of the gold standard NPS results.

## 3. Results

600 salivary samples were included in our study, and 5 of these 600 (0.8%) salivary samples were invalid. The results of the salivary sample were compared with the NPS sample results (Table 1).

The sensitivity detected was 85.34%, specificity was 95.04%, positive predictive value (PPV) was 91.67%, negative predictive value (NPV) was 91.03%, and the measurement agreement (kappa coefficient) was 0.797 (*p* < 0.001) when compared to the gold standard NPS results. The mean Ct value for saliva samples was 11.29 ± 15.21, and the mean for NPS samples Ct value was 10.93 ± 13.55. The difference was not found to be statistically significant (*p* value = 0.433). The correlation between the Ct values of saliva and NPS was found to be 0.692 with a significant *p* value < 0.001.

Out of these 600 samples, 258 random samples were processed by the RT-qPCR RNA extraction-free method using the Thermo Fisher Applied Biosystems kit, of which 27 salivary samples were found to be invalid. The results of the salivary sample were compared with the standard NPS sample (Table 2).

For comparison of the RT-PCR kits, 258 samples that were processed with the Thermo Fisher Kit were matched with their reports when processed using the BGI RT-PCR kit. Of these matched samples, 4 samples were found to be invalid.  Table 3 shows the results of the matched 258 salivary and NPS samples using the BGI kit (Table 3).

The sensitivity, specificity, PPV, NPV, and the percentage of agreement (kappa coefficient) were calculated for both the kits and compared. There was statistically significant difference between the two kits in terms of sensitivity, PPV, agreement percentage, and the percentage of invalid results (Table 4).

The mean Ct values of the saliva and NPS samples were compared in both the kits (Table 5). There was no significant difference in the Ct values of salivary and NPS samples in both the kits. However, there was better correlation of 0.607 (*p* < 0.001) between the Ct values of salivary and NPS samples when the BGI kit was used compared to Thermo Fisher kit, which had a correlation value of 0.472 (*p* < 0.001).

The article "Evaluation of RNA Extraction-Free Method for Detection of SARS-CoV-2 in Salivary Samples for Mass Screening for COVID-19" was published in 2021. Journal: Biomed Res Int.

## 4. Discussion

The study showed that the saliva RT-qPCR RNA extraction-free method has high sensitivity and specificity and is comparable to the gold standard nasopharyngeal swab (NPS). Studies reported earlier have shown similar results, where the sensitivity of saliva samples in detecting SARS-CoV-2 ranges from 73% to 91% and the specificity ranges from 97% to 98.9% [18–20].

In our study, the PPV (91.6%) and NPV (91.03%) were high for direct RNA extraction-free method of saliva testing, and similar results have been reported in other studies [18, 20].

The agreement between the results of saliva and NPS samples was good based on kappa coefficient. The values were similar to other studies that have demonstrated 0.68 to 0.85 kappa coefficient on agreement of salivary samples with the nasopharyngeal swabs [18, 21]. Thus, this study demonstrates that even with the RNA extraction-free method, the result agreement was high between salivary and NPS samples.

However, in this study, we observed that there were variations in the sensitivity and specificity in the direct RNA extraction-free method based on the RT-qPCR kit used. The Thermo Fisher Applied Biosystems kit showed higher sensitivity, PPV, and NPV, whereas the BGI kit showed higher specificity and better agreement (kappa coefficient) between the results of saliva and NPS samples.

In the BGI kit, the mean Ct values of both saliva and NPS were low compared to the mean Ct values of saliva and NPS samples when the Thermo Fisher Applied Biosystems kit was used. Both the kits did not show any statistically significant difference in Ct values between the saliva and the NPS samples. Similarly, studies have reported that there was no significant difference in the Ct values of saliva and the NPS samples, although other studies that have also reported significant difference in the Ct values of saliva and NPS samples [22, 23]. This difference in reported Ct values might be because the saliva viral load declines more rapidly than NPS viral load after initial two weeks of infection, as earlier studies have shown [24].

This study also observed significant correlation between the Ct values of saliva and NPS samples. This correlation was better observed with the BGI kit; similar significant correlations were reported in other studies [25].

From the results obtained, our study found that the drawback of the Thermo Fisher Applied Biosystems kit was the number of invalid reports, which was significantly higher than the BGI kit. This might be due to the fact that it is a multiplex assay, and hence, the presence of impurities or inhibitors in body fluids interferes with the assay [26].

The article "Evaluation of RNA Extraction-Free Method for Detection of SARS-CoV-2 in Salivary Samples for Mass Screening for COVID-19" was published in 2021. Journal: Biomed Res Int.

In the RNA extraction-free method, 3.9% and 1.2% of the patients with a negative NPS had a positive saliva sample result using the BGI kit and the Thermo Fisher Applied Biosystems kit, respectively. Other studies have also reported similar results where saliva samples showed higher detection rates at controlled conditions [21, 27]. This variation in results might be due to preanalytical factors affecting the quality of the NPS samples, which include the skill of the trained healthcare professional, the technique used, transport media, temperature control, and storage conditions [13]. The effect of these preanalytical factors is less pronounced in the saliva sample if 1-hour fasting is strictly adhered to by participants.

Hence, this study shows that saliva can be a reliable alternative sample type for SARS-CoV-2 testing. Similar studies have shown saliva to be a reliable sample even without the RNA extraction process [28]. As the sensitivity and the PPV of the saliva sample is high and comparable to the NPS samples, this method can be highly useful in identifying patients early and isolating them to limit spread. This is particularly true given the ease of collection and lack of trained personnel required by the saliva method.

During the current pandemic where mass testing is mandated, the RNA extraction-free method of saliva sample SARS-CoV-2 testing is time-saving and precludes the need for specific collection devices, transport media, and skilled personnel. This can considerably reduce the burden on the healthcare industry and staff. Moreover, because manufacturing and transport of goods have taken a hard hit and become more limited in the current crisis, these simple techniques enable testing of low volume and minimally processed sample that is not affected by the supply chain constraints [15].

## 5. Strengths and Limitations

The strength of this study is that it not only evaluates the RNA extraction-free method for molecular testing of SARS-CoV-2 of salivary samples but also validates and compares different RT-qPCR kits for extraction-free method using saliva sample. Not many studies have evaluated these.

A limitation of this study is that the study did not consider the number of days the patient has been infected or symptomatic in analysis, as the viral load in the saliva varies with the stages of infection, which might have affected the results of the study.

The article "Evaluation of RNA Extraction-Free Method for Detection of SARS-CoV-2 in Salivary Samples for Mass Screening for COVID-19" was published in 2021. Journal: Biomed Res Int.

## 6. Conclusion

This study concludes that the RNA extraction-free method for molecular testing of SARS-CoV-2 in salivary samples serves as an effective alternative for COVID-19 testing. It is important to note that the nature of salivary sample collected, the method of extraction, and RT-qPCR kit used can all influence the results. Saliva collection is simple with no specialized devices needed for collection, and the extraction-free method saves time, effort, and cost, which would infer that this combination is beneficial for large-scale use for combating the COVID-19 pandemic. This is because it enables mass testing and quick, early reporting to control disease spread more efficiently. Thus, despite the limitations, the RNA extraction-free method for molecular testing of SARS-CoV-2 in salivary samples can be broadly implemented as an alternative for SARS-CoV-2 detection and public health purposes.

## Figures and Tables

**Figure 1:** Process of RNA extraction-free method for molecular testing of SARS-CoV-2.

**Table 1:** Comparison of results of salivary sample with the results of standard NPS using the BGI RT-PCR kit (*n* = 595).

NPS sample (BGI kit)		Positive	Negative	Total
RNA extraction-free method for saliva (BGI kit)	Positive	198	18	216
	Negative	34	345	379
	Total	232	363	595

**Table 2:** Comparison of results of salivary sample with the results of standard NPS using the Thermo Fisher RT-PCR kit (*n* = 231).

NPS sample (Thermo Fisher Applied Biosystems kit)		Positive	Negative	Total
RNA extraction-free method for saliva (Thermo Fisher Applied Biosystems kit)	Positive	200	3	203
	Negative	2	26	28
	Total	202	29	231

**Table 3:** Comparison of the matched salivary samples processed through the BGI kit with the gold standard NPS results (*n* = 254).

NPS sample (BGI kit)		Positive	Negative	Total
RNA extraction-free method for saliva (BGI kit)	Positive	109	10	119
	Negative	19	116	135
	Total	128	126	254

**Table 4:** Compares the parameters between the BGI and Thermo Fisher kit.

Parameters	RNA extraction-free direct method (BGI) *n*-258	RNA extraction-free direct method (Thermo) *n*-258	*p* value
Sensitivity	85.15	99.01	< 0.001
Specificity	92.06	89.65	0.674
PPV	91.59	98.52	< 0.001
NPV	85.92	92.86	0.317
Kappa agreement %	74.8	58.3	<0.001
Invalid results	4/258 (1.5%)	27/258 (10.5%)	<0.0001
False positive results	10/254 (3.9%)	3/231 (1.2%)	0.071

**Table 5:** Comparison of Ct values between the saliva and NPS samples.

Method	Sample	Mean ± SD	*p* value	Correlation	*p* value
BGI kit	Saliva	14.19 ± 15.66	0.632	0.607	<0.001
	NPS	13.80 ± 13.43			
Thermo Fisher kit	Saliva	20.52 ± 12.79	0.343	0.472	<0.001
	NPS	21.24 ± 10.05			

## Data Availability

The data is available with the author, Dr. Sally Mahmoud, Director of Biogenix G42 Healthcare Laboratory and will be produced on request.
